# Effects of Modified Jianpi Qushi Heluo Decoction on Scores of TCM Syndromes, 24 h Urinary Albumin, and Plasma Albumin in IMN of Spleen-Kidney Qi Deficiency

**DOI:** 10.1155/2022/6061709

**Published:** 2022-07-11

**Authors:** KaiPi Wu, HongAi Yin, AnMin Du

**Affiliations:** ^1^Department of Basic Medicine, Changde Vocational and Technical College, Changde, Hunan 415000, China; ^2^Department of Nephrology, No. 1 Traditional Chinese Medicine Hospital of Changde City, Changde, Hunan 415000, China

## Abstract

**Objective:**

To explore the effects of modified Jianpi Qushi Heluo decoction on scores of TCM syndromes, 24 h urinary albumin (UA), and plasma albumin (Alb) in idiopathic membranous nephropathy (IMN) of spleen-kidney qi deficiency.

**Methods:**

A total of 84 patients with IMN of spleen-kidney qi deficiency type admitted to the hospital were enrolled between November 2019 and September 2021. According to the random number table method, they were divided into the observation group (42 cases) and control group (42 cases). The control group was treated with routine Western medicine, while the observation group was additionally treated with modified Jianpi Qushi Heluo decoction. All were continuously treated for 2 months. The clinical curative effect between the two groups was compared. Before and after treatment, scores of TCM syndromes, biochemical indexes (24 h UA, plasma Alb, serum triglyceride (TG), and serum cholesterol (TC)), and T lymphocyte subsets (Th1, Th2, Th1/Th2, and Th17) were compared between the two groups. The occurrence of adverse reactions in both groups during treatment was recorded.

**Results:**

The difference in the total response rate of treatment between the observation group and control group was not statistically significant (90.48% vs. 73.81%) (*P* > 0.05). After 2 months of treatment, scores of TCM syndromes in the observation group were significantly lower than those in the control group, levels of 24 h UA, TG, and TC were significantly lower than those in the control group, and Alb was significantly higher than that in the control group (*P* < 0.05). After 2 months of treatment, levels of peripheral blood Th1 and Th17 in the observation group were significantly lower than those in the control group, while Th2 and Th1/Th2 were higher than those in the control group (*P* < 0.05). The difference in incidence of adverse reactions between the observation group and control group was not statistically significant (4.76% vs. 14.29%) (*P* > 0.05).

**Conclusion:**

The modified Jianpi Qushi Heluo decoction can reduce UA, increase Alb, and improve clinical symptoms and immune function of patients with IMN of spleen-kidney qi deficiency.

## 1. Introduction

The greater the proteinuria, the greater the long-term risk for renal failure. In addition, patients who have membranous nephropathy with nephrotic syndrome have significant morbidity and mortality, in particular related to thromboembolic and cardiovascular complications. There is no specific treatment for membranous nephropathy. Supportive care with the use of diuretics and angiotensin-converting enzyme inhibitors in combination with the angiotensin II receptor blocker is recommended, but these agents have only a limited effect. If the early treatment of kidney disease is not timely, it will cause end-stage renal disease, which will seriously affect the physical and mental health and life safety of patients. Conventional Western medicine treatment of IMN has a long cycle and large drug toxicity and side effects, and the patient's compliance with treatment is low. In addition, the individual differences of patients are large, resulting in poor efficacy [1]. Therefore, it is necessary to find new safe and effective treatment methods. Traditional Chinese medicine believes that IMN of spleen and kidney qi deficiency is caused by factors such as improper diet, fatigue, wind pathogens, water-dampness, and other factors, resulting in dysfunction of zang-fu organs, deficiency of the spleen and kidney, and internal accumulation of dampness and heat, which in turn leads to poor operation of Sanjiao [2]. Therefore, the treatment of this disease should mainly focus on invigorating the spleen and kidney and promoting water and stasis. The formula of strengthening the spleen and removing dampness and collaterals has the functions of strengthening the spleen and nourishing qi, removing dampness and collaterals [3]. Previous studies have shown that traditional Chinese medicine treatment has great advantages in improving clinical symptoms and renal function in patients with IMN [4]. However, there are few clinical reports on the effects of Jianpi Qushi and Luo Fang on the treatment of spleen-kidney qi deficiency type IMN. In view of this, this article aims to explore and analyze the effects of Jianpi Qushi and Luo Fang on TCM syndrome scores, 24 h urinary albumin (UA), and blood plasma albumin (Alb) in the treatment of spleen-kidney qi deficiency type IMN.

## 2. Materials and Methods

### 2.1. General Information

A total of 84 patients with IMN with spleen-kidney qi deficiency type who were admitted to our hospital from November 2019 to September 2021 were selected. Inclusion criteria were as follows: (1) diagnostic criteria: in line with Western medicine IMN diagnostic criteria [5], renal biopsy pathology was grades I and II. (2) TCM diagnostic criteria [6]: syndrome type was spleen-kidney qi deficiency type, main syndrome: waist muscle soreness, fatigue, and foamy urine; secondary symptoms: frequent urination and loose stools; tongue fragrance: thin tongue coating, pale red tongue; and pulse: thin pulse. (3) This study was approved by the hospital ethics committee, and the patients and their families gave their informed consent to this study. Exclusion criteria were as follows: patients with drug allergy in each other, patients with severe liver and kidney dysfunction, patients with mental illness, patients with severe immune organ abnormalities, and patients with infection. They were divided into the observation group and control group by the random number table method, 42 cases in each group. In the observation group, there were 29 males and 13 females, aged 42–60 years, with an average of (51.45 ± 2.14) years, and the course of disease was 4–13 months, with an average of (8.50 ± 1.60) months; in the control group, there were 31 males and 11 females. The age ranged from 42 to 60 years old, with an average of (51.24 ± 2.36) years, and the disease duration was from 4 to 13 months, with an average of (8.26 ± 1.71) months. There was no significant difference in baseline data such as gender, age, and course of disease between the two groups (*P* > 0.05).

### 2.2. Treatment Methods

Both groups were given a low-salt and low-fat diet, and the daily protein intake was controlled at 1–1.2/kg; blood pressure was maintained at 125/75 mmHg with ACEI and ARB; patients with elevated triglyceride (TG) using fibrates. Using fibrates, patients with elevated cholesterol (cholesterol, TC) use statins; if the patient's plasma albumin (Alb) < 20 g/L, use aspirin enteric-coated tablets (manufacturer: Chenxin Pharmaceutical Co., Ltd., approval number: National Medicine Zhunzi H20113013, specification: 100 mg × 60 tablets) 1 tablet/d; patients with hypercoagulopathy are treated with low molecular weight heparin 5000 IU subcutaneous injection and other conventional treatments.

The control group was given cyclosporine soft capsules (manufacturer: Huabei Pharmaceutical Co., Ltd., approval number: H10960009, specification: 25 mg × 50 capsules) on the basis of conventional treatment. The starting dose was 12–15 mg (kg) d), gradually reduce the dose after 1-2 weeks, reduce the initial dose by 5% every week, and maintain the dose of about 5–10 mg (kg/d).

On the basis of the control group, the observation group was combined with the addition and subtraction treatment of Jianpi Qushi and Luo Fang. Drug composition: 30 g of raw *Astragalus*, 15 g each of Atractylodes Rhizoma, lotus leaf, Su Ye, and white peony root, 10 g of licorice, and 20 g each of Fangji, *Angelica sinensis*, and Fangfeng. Dialectical addition and subtraction: add aconite, cinnamon stick, and dried ginger for those with yang deficiency; add *Coix* seed and *Pinellia* for those with damp-heat; add wax gourd peel and red bean for those with obvious edema; add forsythia, honeysuckle, and dandelion for those with obvious heat toxicity. For those with blood stasis syndrome, add *Angelica* and peony. Take 200 mL of water in simmer, 1 dose/d, in the morning and evening after meals. Both groups were treated continuously for 2 months.

### 2.3. Methods

#### 2.3.1. Criteria for Judging Efficacy

After 2 months of treatment, the clinical efficacy of the patients was evaluated. Complete remission: the patient's renal function returned to normal, the urine protein quantitative ≤0.3 g/d, and the symptoms of edema proteinuria, hyperlipidemia, and other symptoms basically disappeared. Partial remission: the patient's edema proteinuria, hyperlipidemia, and other symptoms and renal function were significantly improved, 0.3 g/d < quantitative urine protein<3.5 g/d; ineffective: patients with edema proteinuria, hyperlipidemia, and other symptoms and renal function did not improve or even worsened, and the quantitative urine protein was ≥3.5 g/d. Total clinical efficacy = complete remission rate + partial remission rate [7].

#### 2.3.2. TCM Symptom Score

1 day before treatment and 2 months after treatment, according to the relevant regulations in the “Guidelines for Clinical Research on New Chinese Medicines” [8], the two groups of patients were evaluated for the symptoms of lumbar muscle pain, fatigue, and foamy urine, with each item ranging from 0 to 4. Higher score indicates more severe symptoms.

#### 2.3.3. Biochemical Indicators

One day before treatment and 2 months after treatment, 3 mL of fasting venous blood was drawn from all patients, left standing for 30 min, and then centrifuged (3000 r/min, 15 min), and upper serum was collected and stored at −40°C for future use. The serum TG, TC, and Alb levels of patients were detected by enzyme-linked immunosorbent assay, and the reagents and kits were purchased from Shanghai Valan Biotechnology Co., Ltd. The 24-hour urine of the patients was collected, and 3 mL was reserved for detection. The AU5800 automatic differentiation instrument (Beckman Coulter) was used to detect the 24-hour UA of the patients. The reagents and kits were matched with the instrument. All operation steps are carried out in strict accordance with the instructions.

#### 2.3.4. Immune Function

The percentages of Th1, Th2, and Th17 in peripheral blood were measured by flow cytometry (Beckman FC500 USA) 1 day before treatment and 14 days after treatment, and the Th1/Th2 ratio is calculated.

#### 2.3.5. Adverse Reactions

The occurrence of adverse reactions in the two groups was observed, including vomiting, nausea, and diarrhea.

### 2.4. Statistical Methods

SPSS 22.0 statistical software was used for data analysis. The count data such as adverse reactions and clinical efficacy were expressed by *n*, %, and the chi-square test was performed to meet the normal distribution and homogeneity of the measurement data such as immune function, biochemical indicators, and TCM syndrome scores. The difference between the two groups was compared by the independent sample *t*-test, and the difference between the groups before and after treatment was tested by the paired *t*-test, and *P* < 0.05 or *P* < 0.001was considered to be statistically significant.

## 3. Results

### 3.1. Comparison of Therapeutic Efficacy between the Two Groups of Patients

The total effective rate of patients in the observation group was 90.48%, and there was no significant difference compared with 73.81% in the control group (*P* > 0.05), as given in Table 1.

### 3.2. Comparison of TCM Syndrome Scores between the Two Groups of Patients

Before treatment, there was no significant difference in TCM syndrome scores such as lumbar muscle pain, fatigue, and foamy urine between the two groups (*P* > 0.05). After treatment, the scores of the patients in the observation group were lower than those in the control group (*P* < 0.05), as given in Table 2.

### 3.3. Comparison of Biochemical Indicators between the Two Groups of Patients

Before treatment, there was no significant difference in 24 h UA, Alb, TG, and TC levels between the two groups (*P* > 0.05). 24 h UA, TG, and TC were lower than those of the control group, and Alb was higher than that of the control group after treatment (*P* < 0.001), as given in Table 3.

### 3.4. Comparison of Immune Function between the Two Groups of Patients

Before treatment, there was no significant difference in Th1, Th2, Th17, and Th1/Th2 between the two groups (*P* > 0.05); after treatment, there was no significant difference in Th2 between the two groups (*P* > 0.05); the observation group's Th17 decreased, Th1/Th2 slightly increased, and Th1 and Th17 and Th1/Th2 were lower than the control group (*P* < 0.05), as given in Table 4.

### 3.5. Comparison of Adverse Reactions between the Two Groups of Patients

During the treatment period, 3 cases of vomiting, 1 case of nausea, and 2 cases of diarrhea occurred in the control group, with an adverse reaction rate of 14.29%, and 2 cases of diarrhea occurred in the observation group, with an adverse reaction rate of 4.76%. There was no significant difference in adverse reactions between the two groups (*χ*^2^ = 4.211, *P*=0.240). Adverse reactions resolved with treatment and over time.

## 4. Discussion

IMN belongs to the categories of “edema” and “chronic kidney wind” in traditional Chinese medicine. After a person reaches middle age and old age, the constitution gradually declines, and the qi of the spleen and kidney gradually weakens. Losing one's place and master and acting recklessly, water and dampness overflows, external prostitution of the skin will cause edema of the limbs, and internal discharge of the viscera will cause pleural effusion, and if the spleen is lacking, the yang will not rise and the essence will sink, and if the kidneys are ischemic, the essence will be lost and leaked out, resulting in proteinuria [9, 10]. This disease belongs to the deficiency of the root and the excess and is based on the deficiency of the spleen and kidney, with damp-heat and congestion as the symptoms. Therefore, treatment should benefit the kidneys, strengthen the spleen, cultivate the roots, promote blood and water to treat symptoms, and captures essence and solid astringency [11]. Therefore, this study investigated the effects of the addition and subtraction of Jianpi Qushi and Luo Fang on TCM syndrome scores, 24 h UA, and Alb in the treatment of spleen-kidney qi deficiency type IMN.

The formula for strengthening the spleen and removing dampness and collaterals was created by Professor Yu Renhuan based on the theoretical guidance of Li Dongyuan's “Yin Fire Theory” and Zhang Zhongjing's “water-qi disease” [12]. The raw *Astragalus* in the prescription is a holy medicine for tonifying qi, which can invigorate the spleen and replenish qi. Atractylodes Rhizoma invigorates the spleen and replenishes qi, dries dampness and invigorates water, and supplemented with *Astragalus*, can tonify qi and solidify the appearance, prevent self-invigorating water, reduce swelling, dispel wind and relieve pain, and is beneficial to enter kidney wind and relieve pain. Disperse dampness, play a role in helping diuresis and exfoliation; lotus leaves clear heat and nourish hair, and Qingyang not only evacuates congestion and edema but also drive away rheumatism and relieve pain. *Angelica* is a blood medicine, combined with lotus leaf, and Fangfeng can regulate qi and blood dredge meridians and collaterals; licorice tonifies the spleen and replenishes qi, clears heat and detoxifies, and reconciles various medicines. Modern pharmacological studies have shown that *Astragalus* and *Atractylodes* have the effects of enhancing immunity and antioxidation. Fangfeng has antibacterial and anti-inflammatory effects; lotus leaf can be used to treat hyperlipidemia and has a positive effect on preventing thrombosis. Fangji directly acts on adrenal glands, enhances the function of adrenal cortex, and plays an anti-inflammatory role. Atractylodes Rhizoma protects the liver and gallbladder and has anticoagulation and antibacterial activities. The combination of various medicines plays a role in strengthening the spleen and nourishing qi, dehumidification, and collaterals.

In this study, the TCM syndrome scores in the observation group were significantly lower than those in the control group, suggesting that the use of Jianpi Qushi and Luofang modified and subtracted treatment is beneficial to relieve the clinical symptoms of IMN patients with spleen-kidney qi deficiency. The reason may be that the prescription of strong spleen dehumidification can boost the spleen, replenish qi, diuretic, exhaust coordination side branches, dialectical medication according to the patient's condition, help prescribe the correct drug, improve the patient's efficacy, and then alleviate the patient's clinical symptoms and lowered TCM syndrome scores.

24 h UA is closely related to the renal function of the patient. When the renal barrier of the patient is damaged, a large amount of protein is filtered from the glomerulus, which increases the protein content in the urine [13]. Alb, as an important protein reservoir in the body, can be decomposed into amino acids for tissue synthesis of various other proteins. When Alb is lacking in blood, it will cause edema [14]. The results of this study showed that the 24 h UA, TG, and TC levels in the observation group were significantly lower than those in the control group, and the Alb levels were significantly higher than those in the control group, suggesting that the treatment of Jianpi Qushi and Luofang prescription is beneficial to improve the level of Alb in IMN patients with spleen-kidney qi deficiency and reduce the level of Alb, 24 h UA, TG, and TC levels. The reason may be that the treatment of strengthening the spleen and removing dampness and the addition and subtraction of Luofang can help to improve clinical symptoms, promote protein synthesis, regulate the abnormal blood lipid metabolism, and improve the microcirculation of the patient's body, thereby reducing the level of UA and increasing the level of Alb, and the diuretic effect of *Astragalus* can reduce the leakage of protein [15], and the use of this prescription can restore the function of the spleen and stomach, clear the sample, and remove the dampness, thereby relieving proteinuria. Previous studies have shown that the T lymphocyte subsets in patients with IMN are disordered and the level of inflammation increases, resulting in increased Th1 and Th17 and decreased Th2 [16]. In this study, Th1 and Th17 in the observation group were significantly lower than those in the control group, and Th1/Th2 in the control group was higher than those in the control group. The spleen-removing dampness and collaterals formula is beneficial to reduce the level of inflammation in peripheral blood, reduce the infiltration of inflammatory cells in the kidneys, reduce kidney damage, and then exert immunosuppressive effects and improve the immune function of patients.

In summary, the addition and subtraction treatment of Jianpi Qushi and Luo Fang is beneficial to relieve the clinical symptoms of IMN patients with spleen-kidney qi deficiency, reduce the level of UA, increase the level of Alb, and enhance the immune function. The disadvantages of this study are that the sample size is relatively small, and the observation time is short, which still needs to be further confirmed by expanding the sample size and extending the observation time.

## Figures and Tables

**Table 1:** Comparison of therapeutic efficacy between the two groups of patients (*n*, %).

Group	Number of cases	Complete relief	Partial relief	Invalid	Overall efficiency
Observation group	42	22	16	4	90.48
Control group	42	17	14	11	73.81
*χ * ^2^					4.041
*P*					0.133

**Table 2:** Comparison of TCM syndrome scores between the two groups of patients ($\bar{\text{x}}$ ± *s*, points).

Group	Number of cases	Psoas soreness		Tiredness		Foamy urine	
		Before the treatment	After treatment	Before the treatment	After treatment	Before the treatment	After treatment
Observation group	42	2.40 ± 0.54	0.67 ± 0.48^*∗*^	2.52 ± 0.59	0.71 ± 0.46^*∗*^	2.19 ± 0.45	0.71 ± 0.30^*∗*^
Control group	42	2.31 ± 0.47	0.95 ± 0.22^*∗*^	2.74 ± 0.63	0.93 ± 0.34^*∗*^	2.33 ± 0.61	1.10 ± 0.48^*∗*^
*T*		0.860	3.537	1.608	2.433	1.215	2.602
*P*		0.392	0.001	0.112	0.017	0.228	0.011

Compared with the group of before treatment, ^*∗*^*P* < 0.05.

**Table 3:** Comparison of biochemical indicators between the two groups of patients ($\bar{\text{x}}$ ± *s*, *n* = 42).

Group	24 h UA (g)		Alb (g/L)		TG (mmol/L)		TC (mmol/L)	
	Before the treatment	After treatment	Before the treatment	After treatment	Before the treatment	After treatment	Before the treatment	After treatment
Observation group	3.55 ± 0.94	1.09 ± 0.27^*∗*^	27.14 ± 2.32	42.55 ± 5.20^*∗*^	6.29 ± 1.26	2.48 ± 0.47^*∗*^	8.67 ± 1.12	3.29 ± 1.08^*∗*^
Control group	3.62 ± 0.91	2.39 ± 0.62^*∗*^	26.80 ± 2.85	37.54 ± 3.35^*∗*^	6.24 ± 1.33	3.31 ± 0.73^*∗*^	8.49 ± 1.03	4.23 ± 1.20^*∗*^
*T*	0.313	12.556	0.585	5.251	0.177	6.255	0.740	3.746
*P*	0.755	<0.001	0.560	<0.001	0.860	<0.001	0.461	<0.001

Compared with the group of before treatment, ^*∗*^*P* < 0.05.

**Table 4:** Comparison of immune function between two groups of patients ($\bar{\text{x}}$ ± *s*, *n* = 42).

Group	Th1 (%)		Th2 (%)		Th17 (%)		Th1/Th2	
	Before the treatment	After treatment	Before the treatment	After treatment	Before the treatment	After treatment	Before the treatment	After treatment
Observation group	37.71 ± 3.22	23.53 ± 3.30^*∗*^	55.07 ± 2.11	58.26 ± 4.16^*∗*^	7.46 ± 1.49	5.15 ± 1.20^*∗*^	0.67 ± 0.11	0.42 ± 0.10^*∗*^
Control group	36.79 ± 1.80	27.36 ± 3.21^*∗*^	54.88 ± 2.31	56.96 ± 3.26^*∗*^	7.37 ± 1.48	6.39 ± 1.02^*∗*^	0.63 ± 0.19	0.48 ± 0.14^*∗*^
*T*	1.611	5.395	0.404	1.588	0.274	5.070	1.096	2.572
*P*	0.111	<0.001	0.688	0.116	0.785	<0.001	0.276	0.012

Compared with the group of before treatment, ^*∗*^*P* < 0.05.

## Data Availability

The data used to support the conclusion of this study are available from the corresponding author upon request.

## References

[1] Choi J. Y., Chin H. J., Lee H. (2020). Idiopathic membranous nephropathy in older patients: clinical features and outcomes. *PLoS One*.

[2] Nietogaán I., Rita C. G., Perez J. V., Ortego-Pérez S., Rodríguez-Mendiola N., Carrasco-Sayalero Á. (2021). Comparison of 3 anti-PLA2R inmmunoassaysfor the diagnosis of idiopathic membranous nephropathy in an european population. A pilot study. *Clinical Immunology*.

[3] Li C., Li P., Guo W. (2020). The optimal anti-PLA2R cutoff for the diagnosis of idiopathic membranous nephropathy: a single-center retrospective study. *The Korean Journal of Internal Medicine*.

[4] Zhang J., Pan S., Li D. (2020). A nomogram for the prediction of renal outcomes among patients with idiopathic membranous nephropathy. *Experimental and Therapeutic Medicine*.

[5] Shi J., Lu Y., Zhang Y. (2020). Traditional Chinese medicine formulation therapy in the treatment of coronavirus disease 2019 (COVID-19). *The American Journal of Chinese Medicine*.

[6] Zhang X., Liu W., Guo F. (2020). Disrupted structural covariance network in first episode schizophrenia patients: evidence from a large sample MRI-based morphometric study. *Schizophrenia Research*.

[7] Parvizi M. M., Fatehi N., Jaladat A. M., Gholampour Z., Shahriarirad R., Erfani A. (2021). Epidemiological factors in patients with dermatologic conditions referring to the clinic of traditional Persian Medicine: a cross-sectional study. *International Journal of Clinical Practice*.

[8] Cosoli G., Spinsante S., Scalise L. (2021). Wearable devices and diagnostic apps: beyond the borders of traditional medicine, but what about their accuracy and reliability?. *IEEE Instrumentation And Measurement Magazine*.

[9] Wu H. H. L., Alozai A., Li J. W. C. (2022). Risk factors of venous thromboembolism in anti-PLA2R-positive and negative primary membranous nephropathy. *Clinical Kidney Journal*.

[10] Bose B., Chung E. Y. M., Hong R. (2022). Immunosuppression therapy for idiopathic membranous nephropathy: systematic review with network meta-analysis. *Journal of Nephrology*.

[11] Jiang H. X., Feng Z., Zhu Z. B. (2020). Advances of the experimental models of idiopathic membranous nephropathy (Review). *Molecular Medicine Reports*.

[12] Lang R., Wang X., Liang Y., Yan L., Shi B., Yu R. (2020). Research progress in the treatment of idiopathic membranous nephropathy using traditional Chinese medicine. *Journal of Translational Internal Medicine*.

[13] Wang R., Wu Y., Zheng B. (2021). Clinicopathological characteristics and prognosis of hepatitis B associated membranous nephropathy and idiopathic membranous nephropathy complicated with hepatitis B virus infection. *Scientific Reports*.

[14] Hou J., Cheng Y., Hou Y., Wu H. (2019). Lower serum and higher urine immunoglobulin G are associated with an increased severity of idiopathic membranous nephropathy. *Annals of Clinical Laboratory Science*.

[15] Dai P., Xie W., Yu X., Sun J., Wang S., Kawuki J. (2021). Efficacy and cost of different treatment in patients with idiopathic membranous nephropathy: a network meta-analysis and cost-effectiveness analysis. *International Immunopharmacology*.

[16] Ma D. H., Yang X. D., Hua Q. J. (2021). Changes and significance of Treg and Th17 in adult patients with primary membranous nephropathy. *Clinical Nephrology*.

